The article "Serum anticholinergic activity and cerebral cholinergic dysfunction: An EEG study in frail elderly with and without delirium" was published in 2008. Journal: BMC Neurosci.

# Serum anticholinergic activity and cerebral cholinergic dysfunction: An EEG study in frail elderly with and without delirium

**DOI:** 10.1186/1471-2202-9-86

**Published:** 2008-09-15

**Authors:** Christine Thomas, Ute Hestermann, Juergen Kopitz, Konstanze Plaschke, Peter Oster, Martin Driessen, Christoph Mundt, Matthias Weisbrod

**Affiliations:** 1 Centre for Psychosocial Medicine, Department of General Psychiatry, University of Heidelberg, Voßstr. 2, 69115, Heidelberg, Germany; 2 Department of Geriatric Psychiatry, Clinic of Psychiatry and Psychotherapy Bethel, Ev. Hospital Bielefeld, Bethesdaweg 12, 33617, Bielefeld, Germany; 3 Bethanien-Hospital, Geriatric Centre of the University of Heidelberg, Rohrbacher Str. 149, 69126, Heidelberg, Germany; 4 Institute of Molecular Pathology, University of Heidelberg, INF 220, 69120, Heidelberg, Germany; 5 Department of Anaesthesiology, Section: Clinical-Experimental Anaesthesiology, University of Heidelberg, INF 110, 69120, Heidelberg, Germany

## Abstract

**Background:**

Delirium increases morbidity, mortality and healthcare costs especially in the elderly. Serum anticholinergic activity (SAA) is a suggested biomarker for anticholinergic burden and delirium risk, but the association with cerebral cholinergic function remains unclear. To clarify this relationship, we prospectively assessed the correlation of SAA with quantitative electroencephalography (qEEG) power, delirium occurrence, functional and cognitive measures in a cross-sectional sample of acutely hospitalized elderly (> 80 y) with high dementia and delirium prevalence.

**Methods:**

61 consecutively admitted patients over 80 years underwent an extensive clinical and neuropsychological evaluation. SAA was determined by using radio receptor assay as developed by Tune, and standard as well as quantitative EEGs were obtained.

**Results:**

15 patients had dementia with additional delirium (DD) according to expert consensus using DSM-IV criteria, 31 suffered from dementia without delirium (D), 15 were cognitively unimpaired (CU). SAA was clearly detectable in all patients but one (mean 10.9 ± 7.1 pmol/ml), but was not associated with expert-panel approved delirium diagnosis or cognitive functions. Delirium-associated EEG abnormalities included occipital slowing, peak power and alpha decrease, delta and theta power increase and slow wave ratio increase during active delirious states. EEG measures correlated significantly with cognitive performance and delirium severity, but not with SAA levels.

**Conclusion:**

In elderly with acute disease, EEG parameters reliable indicate delirium, but SAA does not seem to reflect cerebral cholinergic function as measured by EEG and is not related to delirium diagnosis.

## Background

Additive long lasting anticholinergic side effects of commonly prescribed drugs have recently gained special interest in neuro-geriatric medicine. They are considered one of the main reasons for cognitive decline [1] and delirium in the elderly. Although delirium is a common cause of morbidity and even mortality in the frail elderly and by this has an enormous impact on health economy as well as on individual quality of life, it remains under-diagnosed in elderly patients and especially in concomitant dementia [2]. Multiple causes underlie confusional states, resulting in a common final pathway of probably stress induced neurotransmission imbalances with a predominant cholinergic deficit [2,3]. Frail elderly are especially at risk because of multimorbidity, polypharmacy, accumulated cerebral pathology and physiological age-related changes. The concept of an anticholinergic burden has been established to highlight overall anticholinergic medication effects that could worsen the often impaired cognitive performance in the elderly, and to mark delirium risk

The anticholinergic burden has been identified using two different approaches.

The first one combines pharmacological knowledge and clinical experience to evaluate the overall central anticholinergic load. [1,4,5] However, mainly peripheral anticholinergic symptoms are screened. The second approach measures the cumulative anticholinergic activity in the peripheral blood utilizing a radio receptor assay developed by Tune in 1980 [6]. This assay detects muscarinic anticholinergic activity in serum samples in comparison to atropine. It has been used to detect global muscarinic anticholinergic properties of various medications [7] and to approve interventions for reducing the anticholinergic burden [8]. Some authors (see [9] for review) found an association of SAA and delirium in various settings, i.e. surgical, ICU- and medical patients [10-12], while some opposing findings exist in oldest old nursing home patients [13]. Cognitive impairment or lower MMSE was associated with higher SAA especially in dementia [9,14,15], depression [16] and community-dwelled elderly [17] but diverging results have also been reported [14,18,19]. It has been presupposed, that this serum assay also reflects the central situation, but this assumption is unproven and has often been questioned [1,20,21]. The CSF-serum-correlation of anticholinergic activity was only reported in two small samples of younger presurgical patients premedicated with central anticholinergics like scopolamine or midazolam [22,23].

The EEG reflects summation potentials of cortical electric activity, modulated by subcortical structures, in an unsurpassed high temporal resolution. The basic EEG alpha rhythm is modulated by cholinergic thalamo-cortical pathways responsible for attention, alertness and vigilance regulation. Inactivity of the arousal system causes a rise of slow activity due to glial influences[24]. Centrally acting anticholinergics such as scopolamine result in occipital rhythm slowing, slow wave increase and decrease of fast activity [25-27], a pattern very similar to the EEG findings in delirium. Because of this distinct pattern, the EEG is still regarded as the gold standard of delirium diagnosis. [26,28] Especially quantitative EEG (qEEG) evaluation has the potential to detect disease- and pharmaco-related powerdensity changes in the different frequency bands [28,29] even in the elderly with and without concomitant dementia.[30,31]

Here we present a cross-sectional and prospective study which aims to investigate the association of anticholinergic burden assessments and EEG parameter in a patient group with high delirium risk: the oldest old suffering acute medical diseases and dementia. We assessed subgroups of these patients including cognitively unimpaired elderly, patients with dementia and patients with additional delirum. We hypothesized that SAA measurement correlates (i) with routine EEG (rEEG) and quantitative EEG (qEEG) parameters and (ii) with functional and cognitive measures. If so SAA would indicate the central cholinergic transmission and would be suitable for the use in delirium screening or prevention as has been recommended[32,33].

## Methods

### Subjects

All patients older than 80 years and admitted to the University of Heidelberg Geriatric Centre, Bethanien Hospital, on Tuesdays and Fridays for the treatment of an acute disease were consecutively recruited between October 2003 and May 2004. 61 patients and, when appropriate, their legal guardians gave written informed consent. The study was conducted in accordance with the Declaration of Helsinki and was approved by the university's ethics review board (No.255/2003). All study examinations were conducted on the third day after admission within a 4 hour time frame to limit fluctuation differences. Data evaluation included age, Barthel Index[34] at admission and discharge, length of hospital stay, delirium associated factors (anemia, cachexia, dehydration, acute infections, oxygen saturation, metabolic disturbances, diabetes mellitus, sensory impairment), the number of medications, number of potentially anticholinergic, "delirogenic" medication (corticoids, antibiotics, psychotropic medication, furosemide [7]) and relevant diseases summarized by the Cumulative Illness Rating Scale (CIRS)[35] (see table 1).

**Table 1:** Patient Group and Subgroup Description

(mean ± SD)	**Cognitively Unimpaired ** n = 15	**Dementia ** n = 31	**Delirium with Dementia ** n = 15	**All patients ** n = 61	**Statistics**
**Age**	86.9 ± 4.0	86.3 ± 4.8	85.3 ± 4.6	86.2 ± 4.5	F(2,58) = 0,46; p = 0,44
**CIRS**	26.6 ± 4.8	30.5 ± 4.4	31.7 ± 5.5	29.9 ± 4.9	F(2,58) = 0,74; p = 0,48
**Dementia type (n)** ** AD/mixed/VaD**	---	19/9/3 61/29/10%	9/5/1 60/33/7%	28/14/4 61/29/8% *	
**Medication amount** (Median, range)	5.1 ± 2.7 (5.0; 1–12)	5.3 ± 2.5 (5.0; 1–10)	5.7 ± 2.3 (6.0; 3–9)	5.4 ± 2.5 (5.0; 1–12)	F(2,58) = 0,23; p = 0,79
**delirogenic medication** (Median, range)	1.6 ± 1.6 (1.0; 0–4)	1.8 ± 1.1 (2.0; 0–4)	2.5 ± 1.4 (2.0; 0–5)	1.9 ± 1.3 (2.0; 0–5)	F(2,58) = 0,20; p = 0,15
Acute Infection	1/7%	7/22%	3/20%	11/18%	H (2,61) = 1.755; p = 0.42
days in hospital	20.5 ± 17.1	15.1 ± 6.8	18.1 ± 7.2	17.2 ± 10.4	F(2,58) = 1,43; p = 0,25
**Barthel **admission	62.5 ± 31.2	33.7 ± 24.3	45.0 ± 18.1	43.9 ± 27.2	**F(2,52) = 6.17; p < 0.005 ** **CU >> D; CU > DD**
**-ADL **discharge	75.8 ± 29.0	47.7 ± 31.7	61.7 ± 25.1	59.0 ± 31.2	**F(2,44) = 3.78; p < 0.05 ** **CU > D**
**IQCODE **(norm < 3.3)	3.1 ± 0.2	4.2 ± 0.6	4.2 ± 0.7	4.2 ± 0.7	**F(2,43) = 3.93; p < 0.03 ** **CU < D, CU < DD**
**Delirium Index** **(range 0 – 21)**	2.5 ± 0.7	6.2 ± 4.0	8.7 ± 4.5	6.4 ± 1.1	**H (2, 46) = 7,15 p =,028 ** **CU < D < DD**
**MMSE **(norm > 28 P)	28.8 ± 1.8	16.7 ± 7.5	14.4 ± 6.0	19.1 ± 8.3	**H (2,61) = 32.52; p < 0.001 ** **CU >> D; CU >> DD**
**SPMSQ **(norm < 2)	0.6 ± 0.9	4.7 ± 2.8	6.4 ± 2.7	4.1 ± 3.2	**H(2,60) = 27.24; p < 0.0001 ** **CU << D, CU << DD**
**SAA in pmol/ml ** (w/o extremes > 2SD)	9.33 ± 4.44 (9.33 ± 4.44)	11.03 ± 6.15 (10.27 ± 4.62)	12.25 ± 10.53 (9.77 ± 4.47)	10.91 ± 7.12 (9.91 ± 4.48)	F(2,57) = 0,71; p = 0,50 F(2,55) = 0,62; p = 0,54

Mean ± SD are shown. AD = Alzheimer Dementia, mixed = AD with vascular pathology, VaD = Vascular Dementia, SAA = Serum Anticholinergic Activity,. CIRS = Cumulative Illness Rating Scale, IQCODE = Informant Questionnaire on Cognitive Decline, SPMSQ = Short Portable Mental Status Questionnaire, MMSE = Mini Mental State Examination, Barthel-ADL = Activities of Daily Living. * n = 46 demented patients ANOVA/Kruskal-Willis statistics and posthoc-testing, with < or > giving the direction of the difference at a significance level of p < 0.01; >> or << specifies direction at a higher significance level of p < 0.001

### Clinical and neuropsychological assessment

A consensus panel, consisting of a geriatric psychiatrist and neurologist and a geriatric medicine specialist, provided diagnosis according DSM-IV criteria. Confusion Assessment Method (CAM)[36,37] was used as a screening tool and diagnosis was based on patient's history, neuropsychological testing, a focused caregiver's interview and the Informed Questionnaire on Cognitive Decline of the Elderly (IQCODE)[38] to ensure diagnostic quality of dementia also. Neuropsychological testing included Mini Mental State Examination (MMSE)[39] and the Short Portable Mental Status Questionnaire (SPMSQ)[40]. Delirium severity was judged by the Delirium Index (DI)[41] The patients were assigned to the following groups according to DSMIV criteria for dementia and delirium: **Patients with delirium and dementia (DD) **(n = 15), **demented patients **without delirium **(D) **(n = 31) and **cognitively unimpaired (CU) **(n = 15).

### SAA Measurements

Venous blood was collected 1 hour before EEG recording and immediately stored at 4°C for 1 hour until centrifugation (7.000 rpm, 10 min). The supernatant was stored at -80°C until SAA levels were determined. We used the radio receptor assay developed by Tune et al [6] where anticholinergic agents in patients' serum compete with tritiated quinuclidinyl benzilate for mACH-receptors obtained from rat forebrain/striatum homogenate. The displacement of 3H-QNB was used to quantify SAA in comparison to an Atropine standard curve. Detection limit was 0.5 pmol/ml, samples were assessed as one batch. Intra-assay accuracy was always between 93 and 109%, intra-assay precision was always better than 9%, inter-assay accuracy ranged between 95 and 105% (5 spiked serum samples over 3 days at 5, 10, 25 and 50 pmol/ml).

### EEG Procedures

EEGs were performed mornings in a shielded, quiet room with artificial light with a computerized 32-channel EEG (Nihon Kohden), 10–20 system including VEOG/HEOG, linked C3C4 as reference, 500 Hz sampling rate, 0.03 Hz and 70 Hz filter settings, impedance below 0.5 kOhm. Patients' vigilance was optimized by using regular alerts (pencil knocking). For spectral analysis 50 artifact-free epochs, each of 2 sec duration, were obtained (minute 5 to 8) in those EEGs without focal abnormalities (n = 49) after semiautomatic artifact reduction, artifact detection using EOG traces and manual removal. Routine EEG was assessed according to clinical criteria by an experienced neurophysiologist blinded to the patients' diagnoses.

Spectral analysis data (real and imaginary components) were evaluated on rereferenced (average reference) EEG using Brain Vision Analyzer software (BrainProducts GmbH, Munich, Germany). FFT data for absolute (aPD) and relative power density (rPD), normalized to 1–20 Hz, were calculated for the parieto-occipital region (averaging O1, O2, O9, O10, P3, P4, Pz, P7, P8) since EEG changes in delirium are most prominent occipitally. AP peak power and peak frequency as well as rPD in 2 Hz-frequency bands (delta 1–3 Hz to alpha2 11–13 Hz) and an aPD-slow wave ratio (A/TD = alpha1+alpha2/theta1+theta2+delta) were obtained and Log10 transformed to minimize skew and kurtosis.

### Statistical analysis

Group differences were examined using univariate ANOVAs and Duncan's post-hoc-tests. EEG and log-transformed qEEG variables were evaluated by repeated measures ANOVAs (group*frequency bands) followed by one-way ANOVAs for each variable separately or by Kruskal-Wallis-ANOVAs. Pearson's correlation coefficients were calculated to evaluate the relation of descriptive variables, EEG parameters and SAA. All statistics were calculated using Statistica 6.0 StatSoft, Inc.

## Results

The 61 elderly (86.2 ± 4.5 years, 74% female) had been admitted because of acute infection (n = 11/18%), falls (13/21%), cardiac or metabolic disease (9/15%), stroke (5/8%), acute mental disorders (6/10%) and other medical conditions. Five EEG recordings could not be evaluated because of technical artifacts.

### Clinical Data

Subgroups did not differ with respect to age, number of diagnoses, medication, delirium risk factors or so-called delirogenic medication (table 1). Cognitive impairment was reflected by MMSE and SPMSQ results (p < 0.001) as well as proxies' IQCODE (p < 0.004). Cognitive impairment was greatest in the delirium group. Delirium Index (DI) demonstrated delirium severity (p < 0.02) No statistical differences were revealed between the delirium plus dementia (DD) and the sole dementia group (D) apart from DI. MMSE and DI correlated in dementia (r = 0.89 and delirium plus dementia (r = 0.78). Cognitive impairment correlated strongly with functional status and functional outcome measured by Barthel-Index (r = 0.55; p < 0.005), but no significant correlations were detected with medication amount, delirogenic medication or overall disease severity (CIRS).

### Serum anticholinergic activity

SAA samples were obtained in 60 patients. In one demented patient no SAA activity could be detected. As table 1 depicts, no differences in SAA-levels were found between the three groups indicating that neither delirium nor dementia is reflected. There was no significant correlation between SAA levels and age, functional decline (IQCODE), medication amount, delirogenic medication use, delirium severity (DI) and overall disease severity (CIRS). Analysis for the group as a whole yielded a modest negative relation between cognitive performance and anticholinergic burden (fig. 1a). Two patients, however, showed extremely high SAA values (> 2SD) and were thus excluded from further evaluation. An 82 year old woman with admission diagnosis of anticholinergic delirium due to amitryptiline medication had 47 pmol/ml; an 87 year old male with acute pneumonia, fever, severe dementia and 10 different medications, 4 of which had anticholinergic properties, showed 33 pmol/ml. After their exclusion, correlation with cognitive impairment (MMSE) was no longer significant. Functional outcome was significantly correlated with SAA (fig. 1b).

**Figure 1:** **Correlation between SAA and cognition and outcome**. Only when extremes (Fig.1a: top, bottom right) were included into calculation, negative correlation with MMSE reached significance. Excluding extremes (bottom, Fig. 1b) reveals significant correlation with functional outcome.

### EEG results

Delirium cases revealed the highest amount of standard EEG pathology, exhibiting occipital slowing (11/13), theta and/or delta excess (11/13–85% resp. 9/13–69%), insufficient or lost reactivity (13/13) and anteriorization (11/13) in EEG, significantly different from CU (p < 0.01). Table 2 depicts significantly slowed EEG basic rhythm in dementia and even more occipital slowing in DD. QEEG showed significant delta and theta1 increase as well as alpha decrease in DD, resulting in lower slow wave ratio (A/TD) values compared to CU. In comparison to demented patients without delirium, significant delta increase and alpha2 decrease in DD were revealed.

**Table 2:** Standard EEG and quantitative EEG parameters

	**Cognitively Unimpaired ** n = 13	**Dementia ** N = 30 (24)	**Delirium with Dementia ** n = 13 (12)	**Statistics**
Background activity Hz mean ± SD at rest	9.05 ± 0.67	7.67 ± 1.53	7.21 ± 1.12	**F(2,54) = 7.60; p < 0.002;** **CU >> D >> DD**
aP-Peak frequency (Hz)	8.50 ± 0.84	7.27 ± 1.44	6.66 ± 1.13	**F(2,46) = 7.30, p < 0.002;** **CU >> D >> DD**
A/TD-ratio	1.05 ± 1.10	0.60 ± 1.00	0.22 ± 1.18	**F(2,46) = 7.84, p < 0.002;** **CU > D >> DD;**
rP-Delta μV^2^/Hz	1.21 ± 0.79	1.68 ± 0.79	2.51 ± 0.92	**F(2,46) = 8.45, p < 0.001;** **CU < D << DD;**
rP-Theta1 μV^2^/Hz	0.62 ± 0.30	1.02 ± 0.44	1.14 ± 0.65	**F(2,46) = 5.98, p < 0.005;** **CU << D << DD**
rP-Theta2 μV^2^/Hz	1.75 ± 9.6	1.77 ± 6.7	1.61 ± 0.55	F(2,46) = 0.20, p = 0.82
rP-Alpha1 μV^2^/Hz	2.08 ± 0.94	1.24 ± 0.76	0.86 ± 0.47	**F(2,46) = 9.35, p < 0.0005;** **CU >> D >> DD**
rP-Alpha2 μV^2^/Hz	0.59 ± 0.29	0.49 ± 0.28	0.32 ± 0.15	**F(2,46) = 4.72, p < 0.02;** **CU >> DD; D > DD**

Absolute Power(aP) values are given for Peak frequency and alpha/theta+delta ratio, frequency bands are given in relative powerdensity values, mean ± Standard deviation, ANOVA statistics and Duncan posthoc-testing, with < or > giving the direction of the difference at a significance level of p < 0.01; >> or << specifying direction at a higher significance level of p < 0.001.

Surprisingly, SAA levels did not correlate with any of the EEG parameters (table 3). Thus, the typical EEG signs of acute encephalopathy depicted in DD (delta increase, alpha2 decrease, A/TD-ratio reduction) did not relate to SAA levels. Also, EEG changes due to dementia as a chronic encephalopathy (peak frequency slowing, theta1 increase) did not correlate with the anticholinergic burden indicator in the group of D or DD (fig. 2).

**Table 3:** Correlations between QEEG and Cognition, Serum Anticholinergic Activity and Functional Outcome

	**aP-Peak frequency**	**A/TD-ratio**	**rP-Delta**	**rP-Theta1**	**rP-Theta2**	**rP-Alpha1**	**rP-Alpha2**
**MMSE (n = 49)**	**r = 0.53** **p < 0,0001**	**r = 0.31** **p = 0.027**	**r = -0.40** **p = 0.004**	**r = -0.55** **p = 0.000**	r = 0.09 p = 0.526	**r = 0.51** **p < 0.0001**	**r = 0.37** **p = 0.010**
**DI (n = 40)**	**r = -0.46** **p < 0,003**	**r = -0.32** **p = 0.04**	r = 0.22 p = 0.18	**r = 0.49** **p = 0.001**	r = 0.09 p = 0.526	**r = -0.36** **p < 0.023**	r = -0.26 p = 0.09
**SAA (n = 47)**	r = 0.20 p = 0.171	r = 0.16 p = 0.280	r = 0.17 p = 0.242	r = 0.27 p = 0.067	r = -0.22 p = 0.137	r = 0.09 p = 0.538	r = 0.01 p = 0.98
**BI-ADL admission (n = 45)**	r = 0.01 p = 0.96	r = -0.06 p = 0.684	r = -0.28 p = 0.065	r = -0.17 p = 0.256	r = 0.22 p = 0.146	r = 0.12 p = 0.437	r = 0.22 p = 0.148
**BI-ADL Discharge (n = 38)**	r = 0.23 p = 0.174	**r = 0.40** **p = 0.012**	**r = -0.39** **p = 0.016**	r = -0.23 p = 0.172	r = -0.14 p = 0.404	**r = 0.46** **p = 0.004**	**r = 0.45** **p = 0.004**

Correlations are given for the whole group without extremes (n = 49). aP/rP = absolute/relative Power, SAA = Serum Anticholinergic Activity, BI-ADL = Barthel Index, DI = Delirium Index; significant results are bold.

**Figure 2:** Correlation between cognition, functional status and qEEG parameters.

In contrast, the aforementioned qEEG parameters correlated with cognition (MMSE) (p < 0.005), revealing a negative correlation with slow wave bands, highest with lower theta, and a positive correlation with alpha bands. Similar correlations were found with the DI that underlined the association of EEG slowing and delirium severity. Functional outcome (Barthel-Index at discharge) correlated highest with both alpha bands (p < 0.05) as is depicted in table 3.

## Discussion

In our prospective, cross-sectional study of SAA, which has been proposed for delirium screening [7,33], we detected substantial SAA levels in frail, often demented, elderly. However, SAA levels revealed to be independent of delirium and dementia diagnoses and did not correlate with cognitive impairment. Nor did we find a correlation with any rEEG or qEEG parameter known to be affected by the central anticholinergic action of scopolamine [25,27], and by delirium [26,28]. At least in oldest-old geriatric inpatients, SAA levels do not seem to reflect the cerebral situation as measured by clinical means and by EEG.

High SAA levels indicated a significant anticholinergic burden detectable in the serum of all subgroups of frail elderly with acute medical conditions, but were not related to delirium and dementia diagnosis. SAA levels reported in the literature were measured with comparable methodology but revealed rather divergent levels [7,9], presumably due to the different populations studied. Our SAA levels of frail elderly were in line with those of other investigations in comparable settings [8,10,14], though some groups found much smaller SAA in quite similar patients [9,11,12] especially in patients without delirium.

In our study, SAA levels did not differ in DD patients and the D or CU subgroups which argues against the hypothesis of a direct relation between delirium and SAA. The two comparable studies reporting a significant SAA difference in delirium [10,12] exhibited several methodological drawbacks. Delirium diagnosis in both studies was based on screening instruments only, without psychiatric evaluation; centrally acting anticholinergic drugs were significantly more common with high SAA and delirium [10,11]; outlier biases occurred [10] and infection was the strongest delirium predictor. As in our study, SAA did not correlate with definite anticholinergic drugs overall.[12] Also, delirium itself did not correlate with an overall anticholinergic burden but with specific centrally active drugs [42]. Endogenous contributions to SAA, related to fever and infection rather than delirium, and probably mediated through stress mechanisms were recently detected[13,22,43]. In animals, stress-induced hyperthermia was found to be modulated by a peripheral cholinergic mechanism [44]. It is therefore hypothesized that stress- and fever related endogenous anticholinergic activity operates in the periphery [22].

In conclusion, SAA must be considered as a conglomerate of anticholinergic properties of endogenous and exogenous origin, which act on peripheral targets and only possibly on the CNS. Our results suggest, that SAA reflects predominantly non-central-acting and medication-independent components in frail oldest old with acute disease.

Typical EEG changes represent the gold standard of delirium diagnosis[26,28,30] and our EEG results are in line with these findings in delirium [28,31] and with dementia studies [26,45]. REEG and qEEG parameters correlated closely with delirium severity and cognitive impairment underlining their relation to cholinergic activation.

EEG again confirms our expert panel based clinical subgroup classification, but neither rEEG nor qEEG parameters correlated with SAA levels. EEG patterns of centrally acting anticholinergics such as scopolamine closely resemble delirium changes in normal [25,27] and demented subjects [46] while peripheral anticholinergics do not exhibit EEG changes [27,29]. Thus, the lack of any correlation of SAA with EEG parameters again gives strong evidence that SAA in our sample of frail elderly does not reflect the cerebral cholinergic situation. We confirmed this recently in a younger sample of various ICU patients[47], where SAA levels were found to be lower, but also did not correlate to delirium and EEG measures.

In our frail elderly population no association was observed between the anticholinergic burden and cognitive deficits, not even in dementia. This finding is contrary to previous studies describing an association of SAA with lower MMSE [17,21,22], restricted in some to demented patients [9,14], or to specific memory tests [16]. Others reported no connection in non-demented elderly [14,19]. Reasons for these discrepancies include: Individual variations due to white matter load [21] and ApoE status [48], which have been shown to influence cognitive performance and cognitive challenge recovery in non-demented elderly. Dose-dependent influences of centrally acting anticholinergics are also probable [14,22] and may have been overlooked. In Chew's sample, e.g., most demented subjects had received lorazepam [9], which was recently reconfirmed by fMRT to impair memory [49] and facilitates delirium transition [50]. On the other hand, as MMSE is a rather crude measure of memory functions, slight differences might have been detectable with more sophisticated tests on working memory and delayed recall in our sample, as anticholinergic medication in general has been proven to influence memory function in a subtler way.[1,5]

However, we did find a moderate correlation of SAA with functional outcome, indicating a negative influence of the anticholinergic burden on functional capacity in D and in acutely ill CU, supporting a former study [18]. In DD correlation was lacking, indicating functional deficits caused by additional mechanisms. Functional impairment may be caused by peripheral side effects like accommodation difficulties, brady- or tachycardia and gate disturbance.[20] On the other hand, peripheral cholinergic pathways have also been described to influence memory performance in mice [51], but this awaits confirmation in humans.

Our study has several limitations. A larger sample size might have clarified the correlation with the patients' daily functions. Additionally, more extensive neuropsychological assessment could evaluate specific but subtle cognitive changes, e.g. memory disturbance. The additional assessment of CSF-AA with SAA and EEG parameters would have strengthened conclusions regarding their association. The correlation of CSF-AA and SAA with individual substances and in different patient samples remains to be assessed. Further studies on the central pharmacodynamics of individual substances and on blood-brain-barrier permeability in the elderly are needed. Finally, our sample did not include delirium patients without a prior cognitive decline. These patients must be studied within a younger patient group with lower dementia prevalence.

## Conclusion

Our naturalistic cross-sectional study in frail elderly used qEEG and thorough clinical delirium diagnosis (expert consensus) to demonstrate for the first time that SAA levels in frail elderly with acute medical conditions are not delirium-related and therefore cannot be reliably applied for delirium prevention or prediction in this relevant group of patients. SAA seems to reflect primarily the peripheral endogenous and exogenous anticholinergic activity that, as animal research indicates, might also influence stress-induced thermoregulation and memory performance. Delirium occurrence is, inter alia, dependent on centrally acting anticholinergic mechanisms.

## Authors' contributions

CT and UH conceived the study, participated in its design and coordination and drafted the manuscript. CT evaluated the standard and quantitative EEGs and performed the statistics. JK and KP developed and processed the SAA assays. PO participated in study design, coordination, data interpretation and manuscript drafting. CM and MD participated in study design, data interpretation and critical manuscript revising. MW participated in study design, coordination, data analysis and interpretation and helped drafting the manuscript. All authors read and approved the final manuscript.
